This article has been retracted.

# Overweight and Cognitive Performance: High Body Mass Index Is Associated with Impairment in Reactive Control during Task Switching

**DOI:** 10.3389/fnut.2017.00051

**Published:** 2017-10-31

**Authors:** Laura Steenbergen, Lorenza S. Colzato

**Affiliations:** ^1^Cognitive Psychology Unit, Leiden University, Leiden, Netherlands; ^2^Leiden Institute for Brain and Cognition, Leiden University, Leiden, Netherlands; ^3^Amsterdam Brain and Cognition, University of Amsterdam, Amsterdam, Netherlands; ^4^Department of Cognitive Psychology, Institute of Cognitive Neuroscience, Ruhr University Bochum, Bochum, Germany; ^5^Institute of Sports and Sport Science, University of Kassel, Kassel, Germany

**Keywords:** cognitive flexibility, adiposity, overweight, body mass index, task switching, binge eating

## Abstract

The prevalence of weight problems is increasing worldwide. There is growing evidence that high body mass index (BMI) is associated with frontal lobe dysfunction and deficits in cognitive control. The present study aims to clarify the association between weight status and the degree of impairment in cognitive flexibility, i.e., the ability to efficiently switch from one task to another, by disentangling the preparatory and residual domains of task switching. Twenty-six normal weight (BMI < 25, five males) and twenty-six overweight (BMI ≥ 25, seven males) university students performed a task-switching paradigm that provides a relatively well-established diagnostic measure of proactive vs. reactive control with regard to cognitive flexibility. Compared to individuals with a BMI lower than 25, overweight (i.e., ≥25) was associated with increased switching costs in the reactive switching condition (i.e., when preparation time is short), representing reduced cognitive flexibility in the preparatory domain. In addition, the overweight group reported significantly more depression and binge eating symptoms, although still indicating minimal depression. No between-group differences were found with regard to self-reported autism spectrum symptoms, impulsiveness, state- and trait anxiety, and cognitive reactivity to depression. The present findings are consistent with and extend previous literature showing that elevated BMI in young, otherwise healthy individuals is associated with significantly more switching costs due to inefficiency in the retrieval, implementation, and maintenance of task sets, indicating less efficient cognitive control functioning.

## Introduction

The prevalence of weight problems is increasing, as more and more people worldwide suffer from overweight and obesity (1). Overweight and obesity are defined as “*abnormal or excessive fat accumulation that may impair health*,” also referred to as adiposity (1). In order to classify overweight or obesity, the body mass index (BMI) is used as an index of weight-for-height in kilograms per square meter (kg/m^2^). A BMI higher than 25 indicates overweight, whereas a BMI equal to or higher than 30 indicates obesity (1). The prevalence of obesity has more than doubled since 1980, with most of the world’s population now living in countries where adiposity (i.e., overweight and obesity) is a more frequent cause of death than underweight (1). The increase in prevalence seems to continue unabated and could be regarded as a modern epidemic (2, 3). Adiposity is a major public health concern as it poses a risk factor for cardiovascular diseases, diabetes, musculoskeletal disorders, and some forms of cancer (1). In addition, adiposity is associated with suicidal tendencies (4), decreased self-esteem and social functioning (5), depression (6, 7), and an increased risk for Alzheimer’s disease (8).

The relative sudden onset of adiposity suggests a relation with changes in our environment. The increased availability of high-caloric food and the reduction in physical activity seem the most important contributing factors (1, 9, 10). But despite these changes in environment, not all individuals get overweight or obesity, that is, some individuals are more prone than others. An explanation for this may be found in individual differences that influence the way in which we interact with the changed environment. Although genetic differences have been found to be related to one’s susceptibility to obesity (11), the genetic pool cannot change to such an extent in only a few decades. Genetic factors and differences in metabolic efficiency are therefore not sufficient in explaining why some individuals tend to gain excessive weight more than others. Although it seems logical therefore to assume that differences with regard to the preference for high-caloric food might explain differences in weight status, it is more likely that an inability to control overeating or binge eating contributes to overweight and obesity (12). Indeed, a recent review by van Meer et al. (13) concluded there is no unequivocal association between food preference and weight status, making it more likely that weight status is related to problems in dealing with food cues and the motivation to eat, rather than differences in preference or pleasure. Insight into cognitive control functions related to overeating and overweight may therefore be important for the development of preventive interventions.

There is growing evidence that higher BMI is related to both structural and functional brain differences. For example, BMI was found to relate linearly to reduced prefrontal metabolism in healthy adults with a BMI between 19 and 38 kg/m^2^ (14) and temporal lobe atrophy in elderly individuals with a BMI ranging from 17 to 38 kg/m^2^ (15). When assigning individuals to groups based on BMI [i.e., BMI < 25 = normal weight, BMI ≥ 25 but <30 = overweight, BMI ≥ 30 = obese, see Ref. (1)], studies report similar results. For example, when looking at individuals across the lifespan, obese individuals, compared to overweight and normal weight individuals, demonstrated reduced whole brain and total gray matter volume (16) and reduced white matter tract integrity (17). In addition, reduced functional connectivity in the default mode and temporal lobe networks was observed in obese compared to normal weight younger adults (i.e., aged 22–29 years) (18). In older adults (aged 70–80 years), obese compared to normal weight, but not overweight, individuals are found to demonstrate lower task-related functional connectivity during finger tapping in the default mode network (19). Altogether, these studies indicate possible underlying mechanisms by which elevated BMI may relate to altered brain functioning and subsequent behavior.

Furthermore, high BMI seems to be associated with chronic low-grade inflammation and with augmented production of pro-inflammatory cytokines (20, 21). Cytokines released at the periphery of the body are known to enhance the production of brain-produced cytokines (22). Interestingly, there seems to be a solid link between the effects of inflammation in the brain and the release of dopamine (DA). Indeed, in a group of rhesus monkeys, the supplementation of Levodopa (DA agonist) compensates for the damaging effect of cytokines on striatal DA release (23). This connection between the effects of inflammation in the brain and the release of DA may account for the detrimental effect of dopaminergic driven cognitive functions observed in obese and overweight individuals. Indeed, overweight and obesity are associated with less responsive DA functioning, less striatal DA-D2/D3 receptor density, and diminished phasic striatal DA signaling (24–27). Using positron emission topography, Volkow and colleagues (14, 28) demonstrated that reductions in baseline prefrontal metabolism were related to decreased memory- and executive performance, often thought to rely on fronto-striatal structures (29), suggesting structural differences associated with elevated BMI are associated with decreased cognitive functioning. Further support for this idea comes from the association between elevated BMI and dysfunctions in executive function across the lifespan (30). More specifically, higher BMI has been associated with poorer inhibitory control as assessed using self-report and behavioral measures in overweight and obese but otherwise healthy individuals across the lifespan (30–35). Although findings are not unequivocal and it has been put forward that behavioral measures may be more adequate than self-report measures for assessing inhibitory control in overweight or obese individuals (33), other studies demonstrate no difference with regard to behavioral inhibitory control as measured by the Stop Signal task (36) and the Stroop task (14). High BMI has furthermore been associated with impairments in memory performance in obese, elderly (i.e., aged 55–88 years), men but not women (37), and impairments in cognitive flexibility as measured by a paper and pencil version of the Stroop paradigm in overweight and obese adolescents (aged 12–17 years) (38). Importantly, dysfunctions in cognitive control (e.g., cognitive flexibility) reflect an impairment in one’s ability to self-regulate a number of mental processes that are needed in order to accomplish task-goals, the importance of which becomes apparent when looking at individuals suffering from such dysfunctions [e.g., in Parkinson’s disease, attention deficit hyperactivity disorder, addiction or obsessive–compulsive disorder, see also Ref. (29)].

According to Cools and D’Esposito (39), cognitive flexibility [i.e., a key cognitive control function (40)] is modulated by striatal DA in a way that it facilitates the updating of information (e.g., about the current task set) in working memory. Indeed, administering the DA-D2 receptor agonist bromocriptine to individuals with low baseline working memory capacity resulted in potentiation of striatal activity and decreased switching costs (41), indicative of enhanced cognitive flexibility (40, 42). In addition, administering tyrosine, the chemical precursor of DA and (nor)adrenalin, enhanced task-switching performance (43). Propranolol, a central and peripheral beta-adrenergic antagonist, did not affect task-switching performance (44), as such contributing to the idea of a key role of DA in task switching. Interestingly, elevated BMI has been associated with both impairments in functional connectivity in the fronto-striatal pathways and DA functioning (8, 14, 18, 19, 24, 25). Hence, given the link between DA pathways and cognitive flexibility, and the link between increases in BMI and DA functioning, the current study focuses on further investigating the relation between BMI and cognitive flexibility.

More specifically, a process-pure measure of cognitive flexibility has been represented by task-switching performance (40, 42). Switching costs are thought to consist of two major components: a preparatory component and a residual component, also referred to as reactive vs. proactive task switching, respectively (45). Using the task-switching paradigm as developed by Rogers and Monsell (46), it is possible to disentangle these components and gain insight in which processes may be affected by elevated BMI. In this paradigm, the sequence of tasks is predictable (i.e., AABBAABB, etc.). The time between the previous response and the upcoming stimulus [i.e., the response-stimulus interval (RSI)] can therefore be considered as preparation interval. Accordingly, when switching from one task to the other, participants make use of this preparation interval to reconfigure the cognitive task set to the demands of the upcoming task. However, the shorter this interval, the less likely the reconfiguration is completed when the next stimulus is presented. Following this, a greater increase in reaction time (RT) on a switch trial (i.e., the switch cost) is usually observed with shorter RSIs, reflecting preparatory switch costs related to processes underlying the retrieval, implementation, and maintenance of task sets [i.e., reactive task switching (46)]. When the RSI is sufficiently long, however, the preparatory component is nearly eliminated (47), but a residual component reflecting inertia or stimulus triggered re-activation of the old task set remains that occurs after stimulus presentation [i.e., proactive task switching; see Ref. (42, 48)]. As the neurobiological and functional neuroanatomical systems related to cognitive flexibility seem somewhat dysfunctional or impaired in overweight individuals, we hypothesize overweight individuals who show impaired cognitive flexibility, as reflected by increased switch costs. Disentangling the preparatory vs. the residual component in relation to overweight may give important insights as to how (decrements in) cognitive control mechanisms are related to overweight, and what preventive measures may focus on. An effect of overweight on the preparatory component would be visible in effects on switching costs when the RSI is short, while an effect on the residual component would be visible on switching costs when RSI is long.

As mentioned earlier, the inability to control excessive food intake (i.e., overeating or binge eating) may be related to less efficient cognitive control (12, 49) and trait impulsiveness (35, 50), but see Ref. (33). We therefore predict overweight individuals, in addition to increased switching costs, to report more symptoms of binge eating and higher trait impulsiveness. In addition, we assessed anxiety [i.e., as measured with the state-trait anxiety inventory (STAI) (51)], depression [i.e., using Beck’s Depression Inventory II (BDI-II) (52)], cognitive reactivity [i.e., using the Leiden index for depression sensitivity-revised (53)], and autistic traits [i.e., using the Autism Quotient (54)], as overweight and obesity have been demonstrated to relate to anxiety and depression (55–57), cognitive reactivity to sad mood (58), and autism (59). Despite BMI being the main classification system for overweight and obesity (1), studies suggest fat percentage, waist circumference, and waist-to-hip ratio may be additional important factors in determining overweight [for a review see Ref. (60)]. For example, increases in BMI may be related to increases in muscle mass rather than fat mass. The other way around, when a person has increased body fat but decreased muscle mass, BMI may not be elevated (61). Therefore, in the current study, we assessed these factors in addition to standard BMI measurements.

## Materials and Methods

### Participants and Design

Participants were 52 healthy adults (12 males) aged 18–26 years (*M* = 20.33, SD = 2.14) who received course credit or a small monetary reward for participation. Using a covert recruitment strategy, potential volunteers were asked to fill in a questionnaire that assessed their general health and other preferences (e.g., religious belief and preferred temperature). Specifically, participants were asked the following questions: (1) What is your age? (2) Do you feel healthy? (3) How tall are you? (4) How much do you weigh? (5) Are you baptized? (6) How often are you going to the mosque or church? (7) How often do you pray? (8) How many hours a week do you play video games? (9) Since what age do you play videogames? (10) Do you have a certain phobia? If so, for what? (11) Do you prefer the heater high or low? (12) Do you work/study better when the heater is high or low? (13) Are you currently taking any medication? (14) Are you or have you been treated by a specialist, including a psychiatrist? (15) Are there any severe psychiatric diseases present in your family history? And (16) Do you use soft- or hard drugs? In addition, all participants were screened using the Mini International Neuropsychiatric Interview [M.I.N.I. (62)]. The M.I.N.I. is a short, structured interview that screens for several psychiatric disorders and drug use, typically used in clinical research (62–64). Participants were only allowed to participate if they met the following criteria: age between 18 and 35, BMI > 18.5, no personal or family history of neurological or psychiatric disorders, no history of substance abuse or dependence, no chronic or acute use of medication, not currently taking part in a weight-loss program, general feeling of being healthy. Following the assessment of BMI, participants were considered to be normal weight (BMI < 25; from now on referred to as the “normal weight group”) or overweight (BMI ≥ 25; from now on referred to as the “overweight group”) according to classification criteria of the WHO (1). BMI measures ranged from 19.6 to 33.0 (*M* = 24.62, SD = 3.44).

### Materials and Procedures

Upon arrival participants read and signed the informed consent, after which they filled out the screening questionnaire. Next, participants filed out the binge eating scale [BES, see Ref. (65)], a 16-item self-report questionnaire that measures the presence of binge eating behaviors. Scores range from 0 to 32, with higher scores indicating more severe binge eating symptoms (66). After filling out these questionnaires, participants first practiced and then performed the task-switching paradigm, which took about 25 min, after which participants completed this session.

In an additional session, participants were weighed and their BMI, percentage bodyfat, and percentage muscle were measured using an OMRON Body Composition Scale Karada Scan. In addition, waist circumference (measured 2 cm above the umbilicus) and hip circumference were measured while participants exhaled and relaxed the abdomen. Finally, participants filled out the following questionnaires.

The autism spectrum quotient [AQ (54)] comprises 50 statements, each of which allows the subject to indicate “definitely agree,” “slightly agree,” “slightly disagree,” or “definitely disagree.” Approximately half the questions are worded to elicit an “agree” response from neurotypical individuals, and half to elicit a “disagree” response. The subject scores one point for each question which is answered either slightly or definitely not neurotypical, leading to a minimum score of 0 and a maximum score of 50. The questions cover five different domains associated with the autism spectrum: social skills, communication skills, imagination, attention to detail, and attention switching/tolerance of change.

The BDI-II (52) is a widely used 21-item multiple-choice self-report questionnaire with high internal consistency [α = 0.91 (52)], which assesses the existence and severity of current (past 2 weeks) depressive symptoms. Participants were presented with items related to symptoms of depression and asked to choose, for each item, the statement that best described how they have been feeling during the past 2 weeks (including the current day). Items are rated on a four-point scale ranging from 0 to 3 in terms of severity. The total score is calculated by adding-up all items; hence, scores range between 0 and 63 [0–13: minimal depression, 14–19: mild depression, 20–28: moderate depression, and 29–63: severe depression (67)].

The Barratt Impulsiveness Scale [BIS-11 (68)] is a 30-item self-report questionnaire to assess trait impulsivity, including impulsive and non-impulsive (reverse scored items) preferences and behaviors. Total scores range from 30 (i.e., low self-reported impulsivity) to 120 (i.e., high self-reported impulsivity). Calculation of these total scores are based on a Likert-type scoring of each item on a scale from 1 (rarely/never) to 4 (almost always/always). Factor analysis by Patton et al. (68) shows that there three independent subscales; eight items assessing attentional impulsiveness (i.e., an impatient tendency reflected by rapid shifts in attention), 11 items comprising motor impulsiveness (i.e., a “reckless” tendency reflected by immediate actions), and 11 items tapping non-planning impulsiveness (i.e., a tendency to ignore long-term consequences of actions and not to plan ahead).

The Leiden Index of Depression Sensitivity—revised [LEIDS-r (53)] consists of 34 items that assess the extent to which dysfunctional cognitions are activated when an individual experiences mild dysphoria. Before answering the items, participants were asked to take a few minutes to imagine how they would feel and think if they were to experience a sad mood and then to indicate the extent to which each statement applied to them on a five-point Likert scale ranging from 0 (i.e., “not at all”) to 4 (“very strongly”), as such higher scores reflecting more cognitive reactivity. The LEIDS-r results in a total score and six subscales assessing cognitive reactivity related to aggression, hopelessness/suicidality, acceptance/coping, control/perfectionism, risk aversion, and rumination on sadness.

The STAI (form Y) is a commonly used measure of trait and state anxiety (51). The STAI consists of 20 items assessing trait anxiety and 20 assessing state anxiety. All items are rated on a four-point scale (e.g., ranging from 1, “almost never” to 4, “almost always”). Scores on both scales range from 20 to 80, with higher scores indicating greater anxiety.

Upon completion of these questionnaires, participants were debriefed and awarded course credit or a small monetary reward for participation. The study conformed to the ethical standards of the Declaration of Helsinki, and the protocol was approved by the local ethical committee (Leiden University, Institute for Psychological Research). All participants were naïve to the purpose of the study and gave their written informed consent.

### Task Switching

The task was adapted from Steenbergen et al. (43) and Colzato et al. (69). At all times, a 10-cm square divided into four quadrants was displayed on the computer screen. Stimuli were presented in white on a black background. Each pair subtended a visual angle of 1.4° both horizontally and vertically. Stimulus location, i.e., the quadrant it was presented in, changed in a clockwise manner across trials. On each trial, a character pair was presented in uppercase in the center of one of the quadrants. When a stimulus pair was presented in one of the upper two quadrants, participants were supposed to perform a letter task, whereas a pair presented in one of the lower two quadrants required a number task. Hence, the display location of the stimuli served as a task cue. Importantly, the order of the tasks was predictable as stimuli were presented in the quadrants clockwise, which implies the task changed predictably every other trial. Depending on the location (i.e., the required task), the relevant character in the pair was either a letter or a number. The second and irrelevant character was either a member of the other category, so that the response afforded by this character was either congruent or incongruent with the task-relevant response, or was drawn from a set of neutral characters. Participants responded using a QWERTY keyboard with their left index finger (on the “C” key) to indicate “even” or “consonant,” or their right index finger (on the “M” key) to indicate “odd” or “vowel.” Consonants were sampled randomly from the set ⟨G, K, M, R⟩, vowels from the set ⟨A, E, I, U⟩, even numbers from the set ⟨2, 4, 6, 8⟩, odd numbers from the set ⟨3, 5, 7, 9⟩, and neutral characters from the set ⟨#, ?, *, %⟩, with the constraint that a character could not be repeated on successive trials. The position of the task-relevant character within a pair was randomly determined on each trial. Stimuli were displayed until a response was registered. Participants received a practice set of two non-switch blocks of 40 trials each to familiarize with the letter and number tasks, respectively. Immediately after, they performed a practice set of nine switch blocks, each with 16 trials, before entering the experimental phase. This consisted of two sets of 15 blocks, each block consisting of 16 trials. The two sets differed with regard to the RSI, in order to be able to disentangle the preparatory and residual component. One block adapted an RSI of 150 ms (i.e., in which switch costs reflect preparatory costs), whereas the other block adapted an RSI of 1,200 ms (i.e., in which switch costs reflect residual costs). The order of the RSIs was randomized across participants.

### Statistical Analyses

Statistical tests were performed using IBM SPSS Statistics 23. A significance level of *p* < 0.05 was adopted for all statistical tests. In case of a significant interaction, *post hoc* analyses were conducted using Fisher’s LSD tests.

#### Participants’ Physical Characteristics

Shapiro–Wilk tests were performed to test for normality assumptions. Separate independent-sample *t*-tests or non-parametric Mann–Whitney *U* tests (i.e., depending on whether or not normality could be assumed) were performed to assess between-group (normal weight vs. overweight) differences in terms of BMI, age, percentage body fat (as measured with the body composition Karada scan), percentage muscle, waist circumference, and waist-to-hip ratio. A Chi-square test was performed to rule out possible differences between low and high BMI groups in terms of gender distribution.

#### Task Switching

The effect of BMI on cognitive flexibility was assessed by submitting mean correct RTs and percentage of errors (PEs) to separate repeated measures analyses of variance (ANOVAs) with task repetition (repetition vs. alternation of task) and RSI (150 vs. 1,200 ms) as within-subject factor and weight group as between-subjects factor. For all participants and for both RTs and PEs, task-switching costs were calculated separately for each RSI by subtracting RTs/PEs on task repetition trials from RTs/PEs on task alternation trials. The first trial of each block was excluded from all analyses.

#### Questionnaires

Shapiro–Wilk tests were performed to test for normality assumptions. Separate independent-sample *t*-tests or non-parametric Mann–Whitney *U* tests (i.e., depending on whether or not normality could be assumed) were performed to assess between-group differences on the AQ total score, BDI total score, BES total score, BIS-II total score and subscales (i.e., attentional impulsiveness, motor impulsiveness, and non-planning impulsiveness), LEIDS-r total score and subscales (i.e., aggression, rumination, risk avoidance, hopelessness, acceptance, and perfectionism), and state- and trait anxiety scores.

## Results

### Participants’ Physical Characteristics

Sample information is shown in Table 1. No significant between-group differences were observed in terms of age, *Z* = −0.363, *p* = 0.717, or gender distribution, χ^2^(*N* = 52) = 0.433, *p* = 0.510. In comparison to the normal weight group, participants in the overweight group were observed to have a significantly higher BMI, *Z* = −6.187, *p* < 0.001, percentage body fat, *t*(50) = −4.194, *p* < 0.001, waist circumference, *t*(50) = −6.261, *p* < 0.001, hip circumference, *t*(50) = −6.158, *p* < 0.001, and percentage muscle, *Z* = −2.224, *p* = 0.026, but no differences were observed for, or waist-to-hip-ratio, *Z* = −1.309, *p* = 0.191 (see Table 1).

**Table 1:** Physical characteristics of the participants, separated for the low and high body mass index (BMI) groups.

	Normal weight	Overweight
*N* [M:F]	26 [5:21]	26 [7:19]
Age (years)	20.38 (0.41)	20.27 (0.44)
BMI (kg/m^2^)**	21.67 (0.25)	27.58 (0.41)
Percentage body fat**	27.75 (1.39)	36.38 (1.52)
Percentage muscle*	31.68 (1.15)	29.00 (1.02)
Waist circumference (cm)**	72.00 (1.21)	83.94 (1.48)
Hip circumference (cm)**	89.81 (1.48)	102.38 (1.40)
Waist-to-hip ratio	0.81 (0.02)	0.82 (0.01)

*SEs are given within parentheses*.

Significant mean between-group difference; *p < 0.05, **p < 0.001.

### Task Switching

Table 2 provides an overview of the relevant outcomes for the RT and PE analyses. Repeated measures ANOVA performed on RTs revealed significant main effects of task repetition, *F*(1,50) = 346.23, *p* < 0.001, $\eta_{p}^{2}=0.87$, and RSI, *F*(1,50) = 79.31, *p* < 0.001, $\eta_{p}^{2}=0.61$: participants responded significantly faster on repetition trials (*M* = 656 ms, SEM = 10.7) than alternation trials (*M* = 878 ms, SEM = 17.3) and when the RSI was long (*M* = 719 ms, SEM = 12.7) than short (*M* = 815 ms, SEM = 15.5). A significant interaction involving these two factors was also observed, *F*(1,50) = 85.51, *p* < 0.001, $\eta_{p}^{2}=0.63$, with switching costs being more pronounced for the short (*M* = 270 ms, SEM = 14.6) than for the long (*M* = 174 ms, SEM = 11.2) RSI. More importantly, a significant three-way interaction involving the factors task repetition, RSI, and group was found, *F*(1,50) = 4.37, *p* = 0.042, $\eta_{p}^{2}=0.08$. Fisher’s LSD *post hoc* tests showed that switching costs differed significantly between normal weight and overweight groups for the short RSI (*p* = 0.038), but not for the long RSI (*p* = 0.66), indicating that the overweight group demonstrates less efficient cognitive flexibility (i.e., more pronounced switching costs), but only for the short RSI (see Table 2 and Figure 1). No significant other sources of variance were observed for the RT analysis, *F_s_* ≤ 1.9, *p_s_* ≥ 0.17.

**Table 2:** Mean reaction times (RTs, in millisecond), percentage of errors (PEs, in percent), and switching costs (alternation–repetition) as a function of weight group (normal vs. overweight), response-stimulus interval (150 ms, short vs. 1,200 ms, long) and task repetition (repetition vs. alternation).

	Normal weight		Overweight	
SOA	150	1,200	150	1,200
**Repetition**				
RTs (ms)	682 (17.6)	624 (15.6)	677 (17.6)	640 (15.3)
PEs (%)	3.7 (0.9)	4.3 (0.6)	5.2 (0.9)	4.0 (0.6)
**Alternation**				
RTs (ms)	925 (29.3)	793 (23.2)	974 (29.3)	820 (23.2)
PEs (%)	8.2 (1.3)	8.5 (1.1)	11.1 (1.3)	8.6 (1.1)
***Switch costs***				
RTs (ms)	243 (20.7)*	168 (15.8)	297 (20.7)*	180 (15.8)
PEs (%)	4.5 (0.8)	4.2 (0.8)	5.9 (0.8)	4.6 (0.8)

*SEs are shown in parentheses*.

Significant group difference; *p < 0.05.

**Figure 1:** Mean switch costs (calculated as the reaction time difference between alternation and repetition trials) as a function of group (normal weight vs. overweight) and the response-stimulus interval (RSI) (150–1,200). SEs of the switch costs are represented by the error bars.

Percentage of error ANOVA revealed only a significant source of variance, namely, a significant main effect of Task Repetition, *F*(1,50) = 105.75, *p* < 0.001, $\eta_{p}^{2}=0.68$, with fewer errors on repetition trials (*M* = 4.3%, SEM = 0.5) than alternation trials (*M* = 9.1%, SEM = 0.7). All the remaining main effects and interactions were not significant, *F_s_* ≤ 3.4, *p_s_* ≥ 0.07.

### Questionnaires

With regard to the AQ, two participants from the overweight group and two participants from the normal weight group missed an answer to a single question (all different items). For these individuals, the missing value was replaced by the mean of that item. One participant from the overweight group did not fill out the AQ and was therefore excluded from the analysis of this questionnaire. Of the 51 remaining participants, the distribution of neurotypicality did not significantly differ between the two weight groups, as the Mann–Whitney *U* test indicated no significant differences with regard to total AQ scores, *Z* = −1.370, *p* = 0.171, see Table 3 for the mean group scores.

**Table 3:** Mean scores on the questionnaires and, when applicable, subscales.

	Normal weight	Overweight
Autism spectrum quotient	14.27 (1.48)	16.48 (1.49)
Beck Depression Inventory II	5.90 (0.88)	10.27 (1.65)
Binge eating scale	9.15 (0.81)	14.16 (1.12)
Barratt Impulsiveness Scale-II		
Attentional impulsiveness	16.08 (0.46)	17.08 (0.61)
Motor impulsiveness	23.12 (0.65)	24.4 (0.69)
Non-planning impulsiveness	20.12 (0.74)	20.36 (0.84)
Total	59.32 (1.59)	61.84 (1.69)
Leiden Index of Depression Sensitivity—revised		
Hopelessness	5.58 (0.94)	6.15 (1.14)
Acceptance	2.54 (0.47)	3.81 (0.69)
Aggression	7.50 (0.77)	9.58 (1.06)
Control/perfectionism	9.03 (0.70)	9.15 (0.72)
Risk aversion	11.23 (0.66)	10.17 (0.95)
Rumination	11.73 (0.82)	12.31 (0.89)
Total	47.62 (2.96)	51.17 (3.94)
State anxiety	34.28 (1.70)	36.33 (2.19)
Trait anxiety	37.35 (1.86)	40.27 (2.50)

*SEs in parentheses*.

With regard to the BDI, one participant from the normal weight group did not fill out the questionnaire and was therefore excluded from the analysis of this score. Of the remaining 51 participants, one participant from the normal weight group had one missing value, which was replaced by the mean of the scale of that participant. Another participant from the normal weight group had two missing values, which were also replaced by the mean of the scale of that participant. Mann–Whitney *U* test indicated the overweight group to significantly differ from the normal weight group with regard to BDI total score distribution, *Z* = −2.282, *p* = 0.022, see Table 3. However, both groups are still classified as having minimal depression symptoms (67).

Concerning symptoms of binge eating, as assessed by the BES, one participant from the overweight group missed 1/4th of the answers and was therefore removed from the data analyses of this scale. With the remaining 51 participants, a significant between-group difference was found with regard to the distribution of the number of binge eating symptoms, *Z* = −3.169, *p* < 0.01, as shown in Table 3, this indicated that the overweight group reported more binge eating symptoms (*M* = 14.16, SEM = 1.12) than the normal weight group (*M* = 9.15, SEM = 0.81).

No significant between-group differences were found on impulsiveness as assessed by the BIS-II with regard to the total score, *t*(48) = −1.084, *p* = 0.284, or the subscales attentional impulsiveness, *t*(48) = −1.314, *p* = 0.195, motor impulsiveness, *t*(48) = −1.351, *p* = 0.183, or non-planning impulsiveness, *t*(48) = −0.214, *p* = 0.831, see Table 3. Analyses were performed on 50 participants, as two participants (one from the normal weight group and one from the overweight group) did not fill out this questionnaire and were therefore excluded from the analyses of this scale.

With regard to the LEIDS-r, subscale scores were computed with the MEAN function and multiplied by the number of items of the subscale. This allows one missing item per subscale, as was the case for three participants (one from the normal weight group and two from the overweight group) who missed one item, for which the missing value was replaced with the average item score of the participant for that particular subscale. Independent samples *t*-tests revealed no significant between-group differences, neither for the LEIDS-r total score, nor for the aggression, control/perfectionism, or rumination subscales all *p_s_* > 0.120, see Table 3, in addition, Mann–Whitney *U* tests indicated no significant differences for the hopelessness, acceptance, or risk aversion subscales, *Z_s_* ≥ −1.284, *p_s_* ≥ 0.199.

Finally, no significant between-group differences were found for the STAI, nor for state anxiety, *Z* = −0.550, *p* = 0.583 and for trait anxiety, *Z* = 0.544, *p* = 0.544, see Table 3 for the mean scores. For the state anxiety score, three participants (one from the normal weight group and two from the overweight group) were missing one answer, these values were replaced by the mean of that scale using the MEAN function and multiplying by the number of items (i.e., 20). With regard to the trait anxiety score, one participant from the overweight group had a missing value for one item, which was replaced by the mean of the scale using the MEAN function and multiplying by the number of items (i.e., 20). Five participants (three from the normal weight group and two from the overweight group) were excluded from the analyses of trait anxiety as they did not fill out the second form of the STAI.

#### Additional Analyses

Given the significant between-group effects with regard to BMI, fat percentage, muscle percentage, waist circumference, hip circumference, task-switching performance, binge eating symptoms, and depression symptoms, we further explored the interrelations between these variables. However, we would like to point out the exploratory nature of these analyses, as these analyses are not based on *a priori* hypotheses.

First of all, given the observed between-group difference with regard to switch costs in the short RSI condition, we computed Spearman’s rho to assess the correlation between BMI and switch costs. BMI was not found to correlate with switch costs in the long or short RSI conditions (ρ = 0.065, *p* = 0.647 and ρ = 0.234, *p* = 0.095, respectively), see Figure 2. Regarding the interrelations between switch costs (in milliseconds or percentage error), impulsivity, binge eating symptoms, and depression symptoms, we found more binge eating symptoms to correlate to more depression symptoms (ρ = 0.372, *p* = 0.008). Although we found neither a between-group differences regarding self-reported impulsivity nor a linear relation between BMI and impulsivity (ρ = 0.139, *p* = 0.334), self-reported impulsivity correlated negatively to switch costs in percentage error when RSI was short (ρ = −0.327, *p* = 0.021). Switch costs measured in milliseconds furthermore correlated to hip circumference when RSI was short (ρ = 0.280, *p* = 0.044) and to fat percentage and negatively to muscle percentage when RSI was long (ρ = 0.281, *p* = 0.043 and ρ = −0.295, *p* = 0.034, respectively). Depression symptoms positively correlated to waist circumference and hip circumference (ρ = 0.344, *p* = 0.013 and ρ = 0.293, *p* = 0.037, respectively), and binge eating symptoms correlated to fat percentage (ρ = 0.305, *p* = 0.030). No other significant correlations were observed (all *p*_s_ ≥ 0.072).

**Figure 2:** Mean switch costs in milliseconds as a function of body mass index (BMI). **(A)** Switch costs calculated as the reaction time (RT) difference between alternation and repetition trials in the short response-stimulus interval (RSI) (150 ms) condition. **(B)** Switch costs calculated as the RT difference between alternation and repetition trials in the long RSI (1,200 ms) condition. **(C)** Switch costs calculated as the difference between the short RSI and long RSI conditions reflecting implementation or preparatory costs *only* due to a time constraint.

With regard to the absence of a linear relation between BMI and switch costs, as pointed out by Horstmann et al. (25), although in their case implicating overweight to obese individuals, the relation between BMI, DA, and cognitive performance does not seem to be linear, but might instead follow a quadratic function. Fitting a quadratic model of BMI and switch costs by means of curve estimation, however, does not result in a significant model, neither when RSI is long (*r*^2^ = 0.108, *p* = 0.061) nor when RSI is short (*r*^2^ = 0.066, *p* = 0.188). Notably, when analyzing the switch costs in the short RSI condition, switch costs actually reflect preparation costs *in addition to* residual costs. When performing repeated measures ANOVA, however, the two RSI conditions are inserted as two levels of one factor. Hence, when looking at main effects or two-way interactions concerning the short RSI only, the other factor (i.e., long RSI) serves as a covariate, which results in short RSI costs reflecting *only* preparatory costs. Although the *post hoc* LSD fished test indicated a significant between-group difference regarding switch costs in the short RSI (in this case reflecting, again, preparation costs *in addition* to residual costs), as mentioned earlier, in order to evaluate the costs only due to time constraints (i.e., speed of implementation) one has to subtract the switch costs in the long RSI condition from the switch costs in the short RSI condition. Fitting again a quadratic function on the resulting variable, this resulted in a significant model [*F*(2,49) = 4.81, *r*^2^ = 0.164, *p* = 0.012], indicating that implementation (i.e., preparatory) costs in relation to BMI indeed follow an inverted U-shaped function. Notably, implementation costs in the overweight group are significantly higher than in the normal weight group, representing the outcome of the three-way interaction resulting from the RM ANOVA [*M*_normalweight_ = 74 ms, SD = 74 ms, *M*_overweight_ = 118 ms, SD = 76 ms, *t*(50) = −2.092, *p* = 0.042].

That being said, current analyses included two obese individuals (BMI = 32.4 and 33.0) in the overweight group, which allows the possibility that observed effects are driven by these individuals demonstrating rather large switch costs in both conditions (see Figure 2). Based on the WHO definition of overweight and obesity, individuals with a BMI ≥ 30 should be considered obese. In order to analyze the effect of being overweight, but not obese, we therefore performed the task-switching analyses excluding the obese individuals.

First of all, we replicate the RM ANOVA effect, demonstrating a three-way interaction between task repetition, RSI, and group for RTs, *F*(1,48) = 5.683, *p* = 0.021, $\eta_{p}^{2}=0.106$, but not percentage error, *F*(1,48) = 0.329, *p* = 0.569, $\eta_{p}^{2}=0.007$. However, Fisher LSD *post hoc* tests indicate no between-group differences regarding the switch costs, neither for the short RSI (*p* = 0.070, *M*_normalweight_ = 242 ms, SD = 94 ms, *M*_overweight_ = 289 ms, SD = 114 ms) nor for the long RSI (*p* = 0.874 *M*_normalweight_ = 168 ms, SD = 60 ms, *M*_overweight_ = 164 ms, SD = 78 ms). Correlation analyses demonstrate, again, that BMI does not show a linear relation with switch costs in the short or long RSI conditions (ρ = 0.165, *p* = 0.251 and ρ = −0.044, *p* = 0.762, respectively). Fitting again a quadratic model with regard to BMI and switch costs, we replicate our findings, again demonstrating no quadratic relation, neither when RSI was short (*r*^2^ = 0.113, *p* = 0.059) nor when long (*r*^2^ = 0.020, *p* = 0.617). Performing this analysis on the costs only due to lack of preparation (i.e., implementation costs) results in a significant model, *r*^2^ = 0.153, *F*(2,47) = 4.234, *p* = 0.020. In other words, higher switch costs in the overweight group are actually due to implementation costs (switch costs when RSI is short–switch costs when RSI is long; *M*_normalweight_ = 74 ms, SD = 74 ms, *M*_overweight_ = 125 ms, SD = 75 ms, *t*(48) = −2.384, *p* = 0.021), which seem positively correlated with BMI if BMI <25 (ρ = 0.265) and negatively correlated if BMI ≥25 but <30 (ρ = −0.345), although both are non-significant (*p* = 0.099 and 0.192, respectively), see also Figure 2C, possibly due to a lack of power because of the low number of participants in both groups (*N* = 24 in the overweight group and *N* = 26 in the normal weight group).

## Discussion

The prevalence of weight problems is increasing, as more and more people worldwide are getting overweight and obese (1). The increased availability of high-caloric food and the reduction in physical activity seem the most important factors contributing to obesity (1, 9, 10). However, these environmental changes cannot explain why some individuals are more prone than others to get overweight. A key factor in explaining these differences seems to be an inability to control overeating or binge eating that some individuals may suffer from (12). The current study aimed at complementing previous research with regard to cognitive control functions related to, and possibly underlying, overeating and overweight (12). That is, the inability to control excessive food intake (i.e., overeating or binge eating) may be related to less efficient cognitive control (12), and trait impulsiveness (35, 50), but see Ref. (33). Specifically, a previous study in adolescents reported increased BMI was related to impaired cognitive flexibility as measured in a paper and pencil version of the Stroop paradigm (38). However, our study is the first to investigate whether this concerns impairments in the retrieval, implementation, and maintenance of the task set (i.e., costs on the preparatory component), or stimulus triggered re-activation of the old task set remains that occurs after stimulus presentation [i.e., costs on the residual component; see Ref. (42, 48)], or both.

In accordance with our hypothesis, we found overweight individuals, as compared to participants with a BMI lower than 25, demonstrated impaired cognitive flexibility as measured in a task-switching paradigm. However, this difference was only found when the RSI was short rather than long, and additional analyses indicated higher switching costs in the overweight group were found to be due to time constraints (i.e., preparatory/implementation) costs, but not residual costs. This implies an impairment in reactive task switching in the overweight group, thought to be due to either the speed of task set retrieval and implementation or the efficiency to maintain the prepared task set, or both (42, 46). In other words, both groups of participants were comparable with respect to the control operations [the reconfiguration of the task set; see also Ref. (69)] but overweight individuals were less efficient (i.e., slower) to produce this result under time pressure. Additional exploratory analyses also indicated that in normal weight individuals, switch costs are driven more by residual costs (as indicated by a smaller difference between the two RSI conditions on average), but as BMI increases in this group, the difference becomes larger as mostly preparation costs increase, as reflected by the found quadratic relation between BMI and implementation costs. For overweight individuals on the other hand, switch costs seem to be driven more by preparation costs (i.e., as reflected by a larger difference between the two RSI conditions) but as their BMI increases, preparation costs mostly decrease and residual costs mostly enlarge (i.e., the difference between the two RSI conditions becomes smaller). Importantly, these effects remained when excluding the two obese individuals in the current sample, stressing the fact that our conclusions with regard to task switching apply to overweight, but not necessarily obese individuals.

In contrast to earlier studies (35, 50) and against expectation, but in accordance with an earlier study by Nederkoorn et al. (33), we did not observe any difference between self-reported trait impulsiveness in overweight individuals as compared to individuals with a BMI lower than 25, even though earlier studies did. We have to be careful interpreting this result, however, as our sample size is rather small, which limiting the power. Nevertheless, in contrast to self-report measures, as also suggested by Nederkoorn et al. (33), behavioral measures of impulsivity (70) may be more adequate in measuring impulsivity in individuals with overweight. That is, self-report measures may be biased due to demand characteristics or lack of self-insight [see also Ref. (71)], although it has also been suggested that overweight-related impulsivity (i.e., impaired inhibition) may be food-specific and not generalize to general inhibition (3), as would fit with the observations of two studies reporting no differences between normal weight and obese individuals with regard to Stroop and stop signal performance (14, 36). Indeed, and converging with the idea of Volkow et al. (12) that overweight may be the result of an inability to control overeating or binge eating, the overweight individuals did report more symptoms of binge eating. It should be noted, however, that we did not assess dietary patterns in the current study. Hence, although our results demonstrate overweight individuals to display more symptoms of binge eating than normal weight individuals, we have no information on the type of food that is eaten. Despite van Meer et al. (13) reporting no association between food preference (i.e., type of food) and weight status, future studies should clarify the role of dietary pattern in the (cognitive) control of overeating.

In addition to impaired proactive task switching and increased symptoms of binge eating, we found overweight individuals to demonstrate higher self-reported depression symptoms. This is in line with previous studies that found BMI was associated with depression (55–57), although both group mean scores reported here would still be classified as minimal depression (67). We found no significant between-group differences with regard to state- or trait anxiety, cognitive reactivity to sad mood, or self-reported behaviors in the autism spectrum. This seems contradictory as previous studies found that overweight and obesity are related to anxiety (55–57), cognitive reactivity to sad mood (58), and autism (59), but may be explained by the fact that our overweight group consisted mainly of individuals with overweight but not obesity.

In addition to BMI, we assessed percentage body fat, muscle percentage, waist circumference, hip circumference, and waist-to-hip ratio in our sample, as these have been proposed additional important factors in determining overweight and obesity [for a review see Ref. (60)]. That is, classifying individuals on the basis of BMI only does not take into account muscle composition, which can contribute to higher weight, and thus BMI. However, muscle composition is not necessarily an index of overweight or obesity. As such, classification on the basis of BMI may underestimate the association between overweight and cognitive control [see also Ref. (31)]. In the current study, we ruled out such a possibility as we found overweight individuals significantly differed from individuals with a normal BMI (i.e., <25) on percentage body fat, waist circumference, hip circumference, and muscle percentage (i.e., the lower BMI group demonstrating a higher muscle percentage), but not age, or gender distribution. Surprising in light of the recommendations by Peeters et al. (60), we found no between-group differences with regard to waist-to-hip ratio. However, previous studies also found waist circumference but not waist-to-hip ratio to be useful for classifying overweight and obesity (72), which is especially important to consider given that our overweight group mainly consisted of individuals with overweight but not obesity. It must be noted, however, that dietary intake prior to the assessment of the above-mentioned characteristics was not assessed, neither were participants instructed to fast. Hence, it is possible that the bioelectric assessments (i.e., fat percentage, muscle percentage) were biased due to, for example, hydration status.

Taken together, our results converge with previous studies suggesting overweight individuals demonstrate less efficient cognitive flexibility, a key cognitive control function (40). The results further suggest these impairments may be a result of difficulty in preparation (due to time pressure) rather than an inability to perform such operations. More research is needed to investigate whether the impairment in reactive task switching is due to the speed of task set retrieval and implementation, or the efficiency to maintain the prepared task set, or both, and to further investigate the non-linear relation between BMI and task-switching costs due to time constraints, as indicated by the exploratory analyses performed in the current study. In addition, despite previous studies demonstrating that higher BMI is associated with chronic low-grade inflammation and with augmented production of pro-inflammatory cytokines, which may account for the detrimental effect of dopaminergic driven cognitive functions observed in obese and overweight individuals (20–23), it remains to be investigated whether the cognitive control deficits and associated neuronal dysfunctions (14, 16–19) observed in individuals with overweight and obesity play a causal role or are instead the consequence of these conditions (12). Furthermore, diet quality and physical activity may influence cognitive control and weight status, and warrant further investigation in relation to the role of cognitive control in overweight and obesity (73, 74). To this end, studies evaluating cognitive control functioning before and after weight loss or gain may provide useful insight. After all, overweight and obesity are preventable (1), and such studies might help to develop effective weight loss- and preventive interventions (49, 75).

## Ethics Statement

The study conformed to the ethical standards of the Declaration of Helsinki, the protocol was approved by the local ethical committee (Leiden University, Institute for Psychological Research). All participants were naïve to the purpose of the study, and gave their written informed consent.

## Author Contributions

LS performed the study, analyzed and interpreted the data, and contributed to writing the manuscript. LC supervised the project and contributed to scientific discussions and manuscript writing. Both authors critically reviewed the content and approved the final version for publication.

## Conflict of Interest Statement

The authors declare that the research was conducted in the absence of any commercial or financial relationships that could be construed as a potential conflict of interest.
